RETRACTED

# Circular RNA circFAT1(e2) Facilitates Cell Progression through the miR-30e-5P/MYBL2 Pathway in Glioma

**DOI:** 10.1155/2023/7418365

**Published:** 2023-02-01

**Authors:** Zengjin Liu, Shewei Guo, Dongming Yan, Yahui Bai, Zhenyu Song, Xianzhi Liu

**Affiliations:** Department of Neurosurgery, The First Affiliated Hospital of Zhengzhou University, Zhengzhou 450052, China

## Abstract

**Objective:**

To explore the mechanism of glioma from MYB family genes from the perspective of the circRNA-miRNA-mRNA regulatory network.

**Methods:**

First, the MYB family genes were analyzed by multiple bioinformatics analyses to identify one gene most associated with glioma. Then, the prognostic value and clinical characteristics of the gene were evaluated by bioinformatics analysis and experiments in glioma cells. Next, the target miRNA and circRNA were predicted and verified by dual-luciferase reporter assays. Besides, the functions of target circRNA in glioma were investigated by CCK-8 and Transwell assays. At last, the relation between the screened MYB gene, miRNA, and circRNA in glioma was identified by rescue experiments.

**Results:**

After expression and Cox and survival analysis of six MYB family genes, MYBL2 was identified as the gene most associated with glioma. Then, we found that MYBL2 expression in primary gliomas was higher than those in other histologies, and it had variable expression according to clinical features. Furthermore, MYBL2 knockdown in glioma cells impairs cell growth, invasion, and migration in functional studies. Then, miR-30e-5p and circFAT1(e2) were identified as targets of MYBL2 by bioinformatics prediction and experimental verification. Finally, the relationship between circFAT1(e2), MYBL2, and miR-30e-5p was elucidated by rescue experiments.

**Conclusion:**

circFAT1(e2) could promote glioma development by regulating MYBL2 and miR-30e-5p, and MYBL2 has diagnostic and prognostic values in glioma.

## 1. Background

Due to malignant alterations in glial cells in the brain and spinal cord, glioma is the most frequent primary brain tumor [1]. The yearly incidence is between 3 and 8 per 100,000 people [2]. Glioma, like other cancers, is caused by a combination of genetic risk factors and toxins in the environment [3]. Neurofibromatosis (type I) and tuberculous sclerosing disease, for example, are established genetic predisposing factors for glioma [4]. Despite the research advance in pathological mechanisms, diagnosis, and surgical and drug treatment, glioma remains intractable cancer. Thus, it is important to further the molecular mechanism study and look for new therapies for glioma [5].

So far, 30 oncogenes homologous to retrovirus oncogenes have been identified in vertebrate cells, and more than 20 of them have been mapped in the human genome. For the convenience of research, oncogenes are temporarily divided into five families according to their structure, gene products, and function similarity, the MYB gene family included. In this family, its members contain MYBL1, MYBL2, MYBBP1A, MYPOP, MYSM1, and others, and presently, they have been focused on the aspect of cancer development. For example, Bayley and colleagues outline the importance of enhanced MYBL2 expression in the development and pathophysiology of BC, as well as potential therapeutic targets for this multifunctional protein to avoid disease recurrence [6]. The relationship between these oncogenes and cancer inheritance, as well as changes in chromosomes, DNA, and genes, in the development of cancer, is still unclear, and scientists are still exploring the mystery.

RETRACTED

The circRNA-miRNA-mRNA regulatory network is the main mechanism that can influence cancer-related gene expression [7]. The main function of circRNA is as a sponge of miRNAs in this network [8]. Yang et al. for example, indicate that circ-ITCH, a circular RNA, inhibits bladder cancer cell migration and proliferation by sponging miR-17/miR-224 and regulating downstream genes, including p21 and PTEN [9]. Han et al. demonstrate that circRNA MTO1 could bind miR-9 as a miRNA sponge, and since p21 was the target gene of miR-9, p21 was indirectly upregulated by circRNA MTO1, thus resulting in the progression of hepatocellular carcinoma [10].

Previous studies have shown that circFAT1(e2) is a novel circRNA derived from exon 2 of the FAT1 gene. In PTC, circFAT1(e2) exerts oncogenic effects by promoting cell invasion and metastasis and is a potential new target for PTC therapy. It is found in gastric cancer that overexpression of circFAT1(e2) inhibits the proliferation, migration, and invasion of gastric cancer cells and is associated with the overall survival of gastric cancer patients. Moreover, miR-30e-5p is a novel cancer-associated miRNA that plays a key role in the progression of different cancers such as nonsmall cell lung cancer, colorectal cancer, and bladder cancer. However, there are few reports on the functional roles of circFAT1(e2) and miR-30e-5p in glioma.

In the present study, we plan to make research on the relations between MYB family genes and glioma from the aspect of the circRNA-miRNA-mRNA regulatory network. Thus, we perform bioinformatics analysis on MYB family genes and glioma to determine the hub gene related to glioma and predict its target miRNA and circRNA. Finally, these findings will unveil the potential mechanism of glioma.

## 2. Materials and Methods

### 2.1. Batch Analysis of MYBL2 Family Genes

The corresponding data of MYBL2 family genes and glioma were obtained from The Cancer Genome Atlas (TCGA) database (https://portal.gdc.com) [11]. Batch expression analysis was used to screen 6 MYBL2 family genes (MYB, MYBL1, MYBBP1A, MYPOP, MYSM1, and MYBL2) for differential expressions in normal, glioblastoma (GBM), and low-grade glioma (LGG) groups. The *P* value, hazard ratio (HR), and confidence interval (CI) were computed using a univariate Cox regression analysis on the 6 genes. Then, to investigate the relationship between their expressions and prognosis, a progression-free survival (PFS) study was carried out (331 glioma patients vs. 331 controls). The worse the prognosis, the higher the expression, which indicates that the gene promotes tumor formation and is otherwise protective. Finally, we selected one gene most related to glioma for the next analysis.

RETRACTED

### 2.2. Prognostic Analysis of MYBL2 in Glioma

The effect of MYBL2 expression on the survival of primary (202 highly expressed groups vs. 202 lowly expressed groups) and recurrent gliomas (127 highly expressed groups vs. 126 lowly expressed groups) was detected. Then, univariate and multivariate analyses were then performed on MYBL2 and several clinical features (age, gender, race, and grade), and the results were displayed by forest plots. The “rms” program was used to create a nomogram and calibration curve based on the aforementioned data to forecast the 1-year, 3-year, and 5-year survival conditions. The nomogram presented a graphical representation of these characteristics, and the points associated with each risk factor could be used to compute the prognosis risk of an individual patient.

### 2.3. MYBL2 Expressions in Different Histologies and Patients with Different Clinical Features

Next, we evaluated the MYBL2 expressions in O (oligodendroglioma), A (astrocytoma), rO (recurrence of oligodendroglioma), rA (recurrence of astrocytoma), AO (anaplastic oligodendro), AA (anaplastic astrocytoma), rAO (recurrence of anaplastic oligodendro), rAA (recurrence of anaplastic astrocytoma), GBM, rGBM (recurrence of glioblastoma) groups, and patients with different clinical features, including grade (WHO II, WHO III, and WHO IV), IDH mutation status (mutant and wildtype), 1p/19q codeletion status (codel and noncodel), age status (<42 and ≥42), and gender (female and male). All the data were acquired from the TCGA database.

### 2.4. Cell Culture and Transfection

The American Type Culture Collection (ATCC) provided U373 and SW1783 (glioma cells), which were kept in RPMI-1640 media (Thermo Fisher Scientific, USA) with 10% FBS (Life Technologies, USA) in a 37°C incubator with 5% CO_2_. circFAT1(e2) overexpression was achieved using the pcDNA3.1 (+) plasmid. Two siRNAs (si-circ1 and si-circ2) targeting the splice junction site of circFAT1(e2) were ordered from Gene-Pharma (Shanghai, China). MYBL2 was knocked down by si-MYBL2 and overexpressed by over-MYBL2 (Gene Pharma, China). Overexpression and knockdown of miR-30e-5p were accomplished using miR-30e-5p mimics and inhibitors (Gene Pharma, China). Lipofectamine 2000 (Invitrogen, USA) was used to transfect the cells as directed.

RETRACTED

### 2.5. Polymerase Chain Reaction-Quantitative Reverse Transcription (qRT-PCR)

Total RNA was extracted using Trizol (Invitrogen, Carlsad, USA) according to the manufacturer's instructions and quantified using spectrophotometry (ND, Wilmington, USA). The reverse transcription was then completed using a reverse transcription kit (TaKara, Dalian, China). Real-time PCR was performed using the TaKara Premix Ex Taq™ II (USA). An iQ multicolor real-time PCR detection system was used to perform RT-qPCR experiments (Bio-Rad, USA). Quantification was done using the 2^–*ΔΔ*Ct^ technique .

### 2.6. Cell Viability Assays

In a 96-well plate, 1 × 10^4^ cells per well were seeded in a 37°C incubator with 5% CO_2_. CCK-8 kit (Beyotime, China) was used to measure cell proliferation 24 hours, 48 hours, 72 hours, and 96 hours after transfection. The absorption wavelength at 450 nm was detected by the reader.

### 2.7. Transwell Assays

After 24 hours of transfection, cells were collected and resuspended in media without serum. Transwell chamber in 24 well plates (8 *μ*m well, BD Biosciences) was utilized to determine cell migration [12]. Matrigel (BD Biosciences, CA) was precoated in the upper well of the Transwell chamber for invasion detection under a 37°C incubator containing 5% CO_2_ for 1 hour. To summarize, a medium containing 10% FBS was introduced to the bottom chamber. And medium free of FBS was put into the upper chamber under a 37°C incubator for 24 hours. The nonmigrated or noninvaded cells were then wiped clean using a cotton swab, while the migrated or invaded cells were washed in PBS before being fixed in 95 percent paraffin and stained with DAPI. Cells were stochastically photographed and counted under a 200× optical microscope of an individual sample.

### 2.8. Dual-Luciferase Reporter Assays

By annealing double-stranded DNA, the wild type (WT) circFAT1(e2), which included miR-30e-5p-specific binding sites, and the mutant fragment, which contained mutant (Mut) miR-30e-5p binding sites, were created. The Lipofectamine 3000 reagents were used for transfection, and the luciferase activity assay was carried out 24 hours later according to the manufacturer's procedure [13].

RETRACTED

### 2.9. Statistical Analysis

GraphPad Prism 19.0 was used to conduct the analysis. ANOVA was used to analyze differences between two or more groups. The possible associations between gene levels and other clinicopathological characteristics were calculated using Fisher's exact test. Kaplan-Meier curves with log-rank test and Cox regression analysis were used to analyze the patients' overall survival. Statistical significance was determined at *P* < 0.05.

## 3. Results

### 3.1. The Findings of MYBL2 Family Gene Analysis in Glioma

As Figure 1(a) shows, MYB, MYBL2, and MYBL1 had the highest levels in the GBM group, whereas MYBBP1A, MYPOP, and MYSM1 had the highest expression levels in the LGG group. In the Cox regression analysis (Figure 1(b)), the results of MYB, MYBL2, MYBL1, MYBBP1A, and MYPOP were significant (*P* < 0.05), while that of MYSM1 was not significant (*P* > 0.05). So, we chose the first five genes for subsequent PFS analysis. The results showed that their higher expressions were usually accompanied by worse survival status (Figures 1(c)–1(g)). Based on the above analyses, MYBL2 was chosen for the next analysis.

### 3.2. MYBL2 Might Be a Standalone Glioma Prognostic Biomarker

In both primary and recurrent gliomas, patients with highly expressed MYBL2 had worse survival than those with lowly expressed MYBL2 (Figures 2(a) and 2(b)).  Figure 2(c) showed the univariate Cox regression for MYBL2 and clinical factors. Multivariate Cox regression analysis indicated that MYBL2 and age might be independent prognostic biomarkers in gliomas (Figure 2(d)). To establish a more reliable prediction method in clinical practice, we constructed a nomogram integrating MYBL2 and age to predict 1-, 3-, and 5-year survival in glioma patients, and the calibration plot for patient survival prediction showed that the predicted results of the MYBL2 prognostic nomogram were in good agreement with the actual results (Figures 2(e) and 2(f)).

### 3.3. Expression of MYBL2 in Diverse Glioma Histologies and Their Relationship to Clinical Characteristics

The greatest level of MYBL2 expression was found in GBM when the expression level of MYBL2 was analyzed in different histologies (Figure 3(a)). The expression level of MYBL2 rose in different WHO grades of glioma as the grade increased (Figure 3(b)). Besides, MYBL2 had a higher expression in the wild type as for IDH mutation status (Figure 3(c)) and noncodel in 1p/19q codeletion status (Figure 3(d)). Also, the expression level of MYBL2 was increased in a group no less than 42 years ole (Figure 3(e)) and females (Figure 3(f)).

### 3.4. The Impact of MYBL2 Knockdown on Glioma Cell Growth and Metastasis

To reveal the role of MYBL2 in gliomas, we first examined the expression of this gene in gliomas, and the data showed that the gene expression was significantly higher in G1 and tumor tissues than in normal controls (Figures 4(a) and 4(b)). MYBL2 expression levels in SW1783 and U373 cells were subsequently decreased by si-MYBL2 (Figures 4(c) and 4(d)). The effect of MYBL2 expression on cell growth was investigated using CCK-8 assays. When compared to the control group, knocking down MYBL2 significantly slowed the growth of SW1783 and U373 cells (Figures 4(e) and 4(f)). Transwell data also showed that the knockdown of MYBL2 weakened the migratory and invasive abilities of glioma cells (Figures 4(g) and 4(h)). Therefore, these results suggested that MYBL2 could promote the development of glioma.

RETRACTED

### 3.5. The Effect of circFAT1(e2) Knockdown on Glioma Cell Growth and Metastasis

The downstream target of MYBL2 was predicted to be miR-30e-5p by TargetScan, miRTarbase, ENCORI, and miRWalk website; and its low expression was detected in glioma (Figure 5(a)). Then, according to the Venn diagram in Figure 5(b), circFAT1(e2) was obtained as the downstream target of miR-30e-5p. To reveal the role of circFAT1(e2) in glioma, we knocked down circFAT1(e2) in SW1783 (si-circ1 and si-circ2, Figure 5(c)) and overexpressed circFAT1(e2) in U373 (Figure 5(d)). circFAT1(e2) was strongly ablated by si-circ1, so it was selected for the following experiments. CCK-8 experiments showed that ablated circFAT1(e2) largely hindered the proliferation of SW1783 and U373 cells, compared with the control group (Figures 5(e) and 5(f)). Transwell analysis showed that reduced circFAT1(e2) also reduced the migratory and invasive abilities of glioma cells (Figures 5(g) and 5(h)). As a consequence, our findings revealed that circFAT1(e2) was an oncogene in the development of glioma.

### 3.6. circFAT1(e2) Regulates Glioma by Targeting miR-30e-5p and MYBL2

Decreased luciferase activity was confirmed in WT-circFAT1(e2) and WT-MYBL2 in the dual-luciferase reporter assay (Figures 6(a) and 6(b)). The expression of MYBL2 was significantly repressed and upregulated in miR-30e-5p and inhibitor-miR-30e-5p, respectively, suggesting that miR-30e-5p was negatively correlated with the expression of MYBL2 (Figure 6(c)). We also investigated whether the miR-30e-5p/MYBL2 pathway was involved in circFAT1(e2) activity in glioblastoma. After circFAT1(e2) was downregulated, qRT-PCR results revealed that miR-30e-5p levels were dramatically raised. However, after transfection with a miR-30e-5p inhibitor or MYBL2, miR-30e-5p was ablated in SW1783 cells (Figure 6(d)). On the other hand, overexpression circFAT1(e2) in U373 cells drastically decreased miR-30e-5p expression. In glioma cells transfected with miR-30e-5p mimics or si-MYBL2, miR-30e-5p levels were recovered (Figure 6(e)). CCK-8 data also demonstrated in Figures 6(f) and 6(g) that transfection of miR-30e-5p mimic or si-MYBL2 vector could partially restore the oncogenic function induced by the overexpression of circFAT1(e2). These data revealed that miR-30e-5p and circFAT1(e2) had a negative relationship and that circFAT1(e2) acted ontogenically via the miR-30e-5p/MYBL2 pathway.

RETRACTED

## 4. Discussion

Although surgery and drug treatment of glioma have made much progress recently, the prognostic status of patients with malignant glioma is deadly poor, mainly due to the rapid proliferation and poor differentiation of glioma, and the presence of drug-resistant cells that are not sensitive to available treatments in gliomas [14]. Therefore, it is important to understand the occurrence and development of glioma. In the article of Lei et al., they suggested miR-24 could promote glioma progression through CDX1/PI3K/Akt signaling pathway, indicating a novel pathway underlying progression in glioma cells and providing a potential target for glioma treatment [15]. Different from this article, we focus on the MYB family genes and glioma, predict the downstream targets, and verify the prediction by bioinformatics analysis and *in vitro* assays to determine the genes with clinical value in glioma.

In this study, we firstly selected 6 genes, MYB, MYBL1, MYBBP1A, MYPOP, MYSM1, and MYBL2, from the MYB family for the bioinformatic analysis. We found that all 6 genes were upregulated in GBM and LGG groups. MYB, MYBL2, and MYBL1 had the highest levels in the GBM group, whereas MYBBP1A, MYPOP, and MYSM1 had the highest expression levels in the LGG group. In the Cox regression analysis, the statistics of MYB, MYBL2, MYBL1, MYBBP1A, and MYPOP were significant (*P* < 0.05), while MYSM1 was not (*P* > 0.05). Therefore, MYB, MYBL2, MYBL1, MYBBP1A, and MYPOP were analyzed by PFS curves, in which their higher expression indicated a worse prognosis, especially MYBL2. Considering all the results, MYBL2 was chosen for the study.

MYBL2 is a member of the MYB family and is involved in cell apoptosis, cell senescence, tumor growth, and other activities as a member of the MYB family [16]. In the G1/S phase, the transcription level of MYBL2 is higher, which can promote the transcription of DNA topoisomerase 11, cyclinB1, and other genes, all of which are involved in the progress of the cell cycle. MYBL2 can also affect cell cycle progression by participating in DNA damage repair and spindle formation [17]. Moreover, MYBL2 can activate antiapoptotic genes such as APoJ and Bcl-2, thus inhibiting apoptosis. MYBL2 is overexpressed in several cancers, including breast cancer, colorectal cancer, and acute myeloid leukemia, according to recent research, and its protein expression level is linked to a poor clinical prognosis.

RETRACTED

Next, we performed bioinformatics analyses on MYBL2 and glioma and observed that MYBL2 could function as an independent prognostic factor in glioma. MYBL2 had a high expression in primary glioma, and its high expression indicated a bad prognosis, no matter in primary glioma or recurrent glioma. Then, by constructing a prognostic nomogram of MYBL2, it demonstrated that MYBL2 had a good prediction in glioma prognosis. Additionally, the expressions of MYBL2 in different histologies and glioma patients with various clinical features were investigated. We also detected the effect of MYBL2 knockdown in glioma cells. The data showed that downregulation of MYBL2 expression in glioma cells SW1783 and U373 inhibited cell proliferation, invasion, and migration. This indicates that MYBL2 functions as a proto-oncogene in glioma. Therefore, MYBL2 may serve as a biomarker and predictive target for glioma.

The circular RNAs (circRNAs) were first discovered in 1979 [18], and they are a sort of small RNA, which forms a covalently closed continuous loop [19]. Following considerable experimental research, the fact that circRNA extensively regulates cellular activities has been revealed. For example, circRNA exerts its biological function as a miRNA sponge to further affect the downstream gene expressions [20]. Meanwhile, with the advance in research on cancer pathogenesis, the key role of circRNA in modulating carcinoma-associated genes by fine-tuning miRNAs in cancer is gradually recognized [21]. circNRIP1, acting as a microRNA-149-5p sponge, mediated the promotion of gastric cancer (GC) development by the AKT1/mTOR pathway [22]. In addition, Li et al. reveal that circRNA-CER, serving as a miR-136 sponge, adsorbs miRNAs, controls MMP13 expression, and takes part in the degradation of ECM in chondrocytes under osteoarthritis [23].

Based on the analysis of public databases, we found that miR-30e-5p was a downstream target of MYBL2, and circFAT1(e2) was a downstream target of miR-30e-5p. Recent studies have shown that miR-30e-5p is dysregulated in several human cancers. For example, the study by Zhang et al. shows that miR-30e-5p may inhibit the growth and invasion of bladder cancer cells by targeting MTDH [24]. The study by Laudato et al. shows that miR-30e-5p inhibits the invasion and metastasis of colorectal cancer by targeting ITGA6 and ITGB1 [25]. circFAT1(e2) (also known as Hsa circ 0001461) is a protein generated from exon 2 of the FAT1 gene, and its roles have been studied in various cancers [26]. Fang et al. demonstrate that circFAT1(e2) is greatly downregulated in GC [27]. Jia et al. have showed that circFAT1 is an important regulator of cancer stemness and antitumor immunity [28]. circFAT1(e2) sets free miR-548 g RUNX1 via the adsorption of miR-548 g [27]. Nevertheless, the mechanism of circFAT1(e2) in glioma remains unclear. In the current study, we observed that circFAT1(e2) levels were also higher in SW1783 and U373 cells than in controls. CCK-8 and Transwell experiments were carried out to uncover circFAT1(e2)'s function and potential mechanism in glioma in SW1783 and U373. As a result, circFAT1(e2) knockdown greatly inhibited cell growth, migration, and invasion. These findings revealed that circFAT1(e2) was an oncogene involved in glioma incidence and progression. In functional studies, it was verified that miR-30e-5p targets circFAT1(e2), and miR-30e-5p was found to be negatively correlated with circFAT1(e2) and MYBL2. Thus, it was concluded that circFAT1(e2) could facilitate glioma by sponging miR-30e-5p and regulating MYBL2.

RETRACTED

Moreover, there are certain limitations of this study that must also be considered. First, these studies were mostly nonrandomized with a small sample size and had issues related to the risk of bias. Second, the results of this study are rarely validated experimentally; thus, the results of this study should be regarded as preliminary results only. Furthermore, the direct correlation between miRNA and mRNA was not assessed on samples from the same patients. In the future, more studies are needed to further investigate the associations described in this analysis.

## 5. Conclusion

Our findings reveal that MYBL2 is increased in gliomas and that overexpression of MYBL2 is associated with poorer survival and prognosis, implying that MYBL2 might be used as an independent glioma prognostic biomarker. Furthermore, circFAT1(e2) exerts an oncogenic role in glioma cells. Mechanistically, circFAT1(e2) can reduce miR-30e-5p, leading to the elevation of MYBL2, thus promoting tumor cell progression. These findings reveal the potential mechanism between circFAT1(e2) and glioma, providing promising diagnostic biomarkers and therapeutic targets in glioma treatment. Although the above results are considered preliminary, they are encouraging.

## Figures and Tables

**Figure 1:** Batch analysis on MYBL2 family genes. (a) Expression analysis of MYB, MYBL2, MYBL1, MYBBP1A, MYPOP, and MYSM1 in three different groups. (b) Forest plot of Cox regression analysis for MYB, MYBL2, MYBL1, MYBBP1A, MYPOP, and MYSM1. (c–g) PFS analysis of genes with significant *P* values (MYB, MYBL2, MYBL1, MYBBP1A, and MYPOP). ^∗∗^*P* < 0.01 and ^∗∗∗^*P* < 0.001.

RETRACTED

**Figure 2:** Prognostic analysis of MYBL2. (a) Survival analysis on MYBL2 expression in primary glioma. The survival rate of high MYBL2 expression was poor. (b) Survival analysis on MYBL2 expression in recurrent glioma. The survival rate of high MYBL2 expression was poor. (c, d) Cox regression study on MYBL2 and clinical variables (MYBL2, age, gender, race, and grade), both univariate and multivariate. (e) In glioma patients, the nomogram predicts 1-, 3-, and 5-year overall survival. (f) The ideal nomogram is represented by the diagonal dashed line on the calibration curve of the OS nomogram model.

**Figure 3:** MYBL2 expressions in different glioma histologies and their relation with various clinical features. (a) MYBL2 expression differences in different histologies. The abscissa is the histology, and the ordinate is the gene expression of MYBL2. (b) MYBL2 expression differences in different WHO grades. The expression level of MYBL2 increased with the increase in grade. (c) MYBL2 expression differences in IDH mutation status. The expression level of MYBL2 in the wild type was higher than that in the mutant type. (d) MYBL2 expression differences in 1p/19q codeletion status. The expression level of MYBL2 in noncodel was higher than that in codel. (e) The expression differences of MYBL2 in age status. The expression level of MYBL2 in patients older than 42 years was higher than that in patients younger than 42 years. (f) MYBL2 expression differences in gender. There was no significant difference in the expression level of MYBL2 in patients of different genders.

**Figure 4:** Downregulation of MYBL2 inhibits the proliferation, invasion, and migration of SW1783 and U373 cells. (a, b) Boxplots, MYBL2 is highly expressed in G1 and tumor tissues. The red ones represent tumor samples, and the blue ones represent normal samples. (c, d) Downregulation of MYBL2 in SW1783 and U373. (e, f) The proliferative capacity of MYBL2 is attenuated in SW1783 and U373 with si-MYBL2. (g, h) The numbers of invading and migrating cells were reduced after the MYBL2 knockdown. ^∗^*P* < 0.05, ^∗∗^*P* < 0.01, and ^∗∗∗^*P* < 0.001.

**Figure 5:** Effects of knocking down circFAT1(e2) on glioma cell proliferation and metastasis. (a) miR-30e-5p is expressed at lower levels in glioma tumors. Brown represents tumor samples, and white represents normal samples. (b) Website prediction of target circRNA of miR-30e-5p. Purple represents ENCORT, yellow represents circbank, and green represents RNAhybrid. (c) circFAT1(e2) knockdown efficiency by si-circ1 and si-circ2 in SW1783. (d) Overcirculation elevated the expression of circFAT1(e2) in U373 cells. (e, f) In comparison to the si-NC group, circ1 silencing decreased the growth of SW1783 and U373 cells. (g, h) The numbers of migrating and invading cells decreased after circFAT1(e2) knockdown. ^∗^*P* < 0.05, ^∗∗^*P* < 0.01, and ^∗∗∗^*P* < 0.001.

RETRACTED

**Figure 6:** circFAT1(e2) targets miR-30e-5p and MYBL2 to regulate glioma. (a, b) The activity of luciferase in cells transfected with the WT plasmid tended to rise, but the mutant group's activity appeared to be unchanged. (c) miR-30e-5p had a negative relation with MYBL2. (d) Si-circ1 enhanced miR-30e-5p expression, while miR-30e-5p inhibitors and over-MYBL2 were able to counteract this. (e) Reduced miR-30e-5p expression was caused by over-circ expression, which was reversed by over-miR-30e-5p and si-MYBL2. (f, g) CCK-8 assays were applied to verify the results in (d) and (e). ^∗^*P* < 0.05, ^∗∗^*P* < 0.01, and ^∗∗∗^*P* < 0.001.

## Data Availability

The datasets used and/or analyzed during the current study are available from the corresponding author on reasonable request.

## Abbreviations

circRNAs: Circular RNAs
IARC: International Agency for Research on Cancer
GC: Gastric cancer
ATCC: American Type Culture Collection
LGG: Lower-grade glioma
GBM: Glioblastoma multiforme
OS: Overall survival
PFS: Progression-free survival.

## Additional Points

*Mini-abstract*. circFAT1(e2) facilitates glioma progression through the miR-30e-5P/MYBL2 pathway, which offers new directions for the therapy of glioma.
